# A Graph Partition-Based Large-Scale Distribution Network Reconfiguration Method

**DOI:** 10.1155/2022/3169065

**Published:** 2022-03-14

**Authors:** Yuanxia Sha

**Affiliations:** Department of Mathematical Sciences, Daqing Normal University, Daqing 163712, Heilongjiang, China

## Abstract

This article focuses on the analysis of large-scale distribution network reconstruction fused with graph theory and graph partitioning algorithms. Graph theory and graph segmentation algorithms have been rushed by many researchers in the fields of medicine, drone, and neural network. It is a newcomer in the field of computer vision, which can not only realize the division in color but also divide it by image data. The distribution network is also indispensable for new energy, electric machines, but the traditional distribution network has many problems, such as not suitable for distributed power access and excessive network loss. To improve the performance of distribution networks and reduce network losses, this paper A multi-division model for distribution network construction and reconstruction is established, and a graph theory-based division algorithm method is proposed to effectively solve the problem of feeder-to-feeder reconstruction during large-scale distribution in distribution networks. Through its superconductivity phenomenon and the characteristics of clustering algorithm division, this paper uses formulas to show its division principle and gives examples of various distribution network reconstruction algorithms to explore which method of improvement can improve the performance of the distribution network and reduce network losses. The number of iterations is also strictly considered, and the value is taken after multiple iterations to reduce the error. Through the distribution network calculation example, the network loss reduction value is obtained, and the distribution network fault repair model is exemplified. The picture is used to briefly describe the process of distribution network reconstruction and find that the faults of the distribution network can be quickly located and isolated through the FTU, and quickly repaired. Finally, in order to reduce the network loss, reduce the load of power flow calculation, and solve the problem of local optimization, a JA-BE-JA optimization algorithm based on large-scale distribution network reconfiguration is proposed. The mixed sampling method is preferred to test the number of divisions in the four states, and the parameters are selected to test the performance of the improved annealing simulation algorithm, and the conclusion is drawn as follows: the improved graph segmentation algorithm has strong robustness, can avoid local optimization of graph data, and can reduce network loss. Compared with traditional distribution network reconstruction methods, the network loss can be reduced to 454.3 KW, which can be optimized by 10.68% compared with the initial network loss.

## 1. Introduction

As a rigorous and scientific theory, graph theory has now been widely used in various fields. The first successful application of graph theory occurred in the 1990s. Some scholars successfully applied it in the research of image segmentation, which attracted the attention and discussion of many scholars at that time. In the development of modern society, the theory of graph theory has also been applied more effectively and broadly, such as texture synthesis, image restoration, and the complicated construction and reconstruction of power distribution networks in modern society. The emergence of graph theory has become extremely significant, which effectively helps in large-scale problems such as distribution networks. Therefore, by establishing a multipartition model for the construction and reconstruction of the distribution network, this paper proposes a partition algorithm based on graph theory to effectively solve the problem of reconfiguration between feeders during large-scale distribution in the distribution network. The proposal of this algorithm greatly reduces the computational pressure in network reconstruction and can effectively arrive at the most reasonable solution based on the global distribution network. Since graph theory itself is a branch subject based on mathematics, the algorithm proposed in the article is a new and effective graph theory algorithm based on rigorous mathematical proofs. In the reconstruction of the distribution network, the image segmentation technology plays an extremely important role. The topology of the network is changed by constantly switching the switch states of the tie switch and the section switch, so as to regulate the flow of power in the entire distribution network. The branch exchange method, optimal flow mode method, genetic algorithm, etc., are all effectively applied in the construction of the distribution network. The improved graph segmentation algorithm can effectively reduce the network loss caused by the operation of the distribution network. In the subsequent reconstruction of the distribution network, graph segmentation algorithms have great research significance.

The purpose of this article is to study the analysis of large-scale distribution network reconstruction fused with graph theory and graph partitioning algorithms and to propose optimization algorithms to reconstruct the distribution network. The algorithms are tested before and after optimization through experiments and applied in the environment of distribution network reconfiguration, collecting the number of edge cuts in the distributed segmentation of 4 image datasets with data sizes ranging from small to large by the JA-BE-JA algorithm based on the BSP-Spark platform. Then, the edge cut numbers of the JA-BE-JA algorithm are collected based on the BSP-PeerSim platform in the same dataset, and they are all collected after 1200 supersteps to ensure the accuracy of the experiment, and the strong robustness of this algorithm and the characteristics of avoiding local optimization are obtained. A 16-bus distribution network is selected for testing, which contains 3 feeder parts, indicating that this algorithm can be applied to large-scale distribution networks and can reduce network losses. At the same time, it also shows that, in dealing with the problem of large-scale distribution network reconfiguration, the optimization algorithm proposed in this paper has a better effect, has a certain guiding significance, and has both theoretical and practical significance.

The improved algorithm designed in this article has a good application prospect in large-scale distribution network reconstruction. Based on the image segmentation method of graph theory-full variational approximation of the Ginzburg–Landau functional of graph clustering, the power flow algorithm of the distribution network reconstruction and the distribution network fault recovery model to perform certain segmentation of the distribution network and the graph theory explanation, the two do have certain commonalities. Then through experiments, the improved algorithm of graph theory and graph segmentation is integrated into the distribution network reconstruction. In order to avoid errors, there are some details in the experiment, such as the choice of encoder and the choice of iteration times. Finally, it is concluded that this graph partitioning improved algorithm can be better applied to a large-scale distribution network environment, and the network loss and robustness are all optimized, which can play a certain guiding role in future development, and it can also be used for reference in other fields.

## 2. Related Work

The application of graph theory and graph segmentation algorithms in various fields has extremely optimistic development prospects, and all fields have never stopped the research and exploration of graph theory and graph segmentation algorithms in order to have a brighter development prospect. Li and Yang paid attention to the adaptive pinning synchronization problem of random complex dynamic network (CDN); based on the algebraic graph theory and Lyapunov theory, they deduced the design conditions of the pinning controller and performed a strict convergence analysis on the synchronization error of probabilistic meaning. Compared with the existing results, due to the use of graph theory, the topology of the random CDN remains unknown [1]. Keown et al. used a selective high-quality data subset from autism brain imaging data exchange (including 111 ASD and 174 typical developmental participants) and several graph theory indicators. They preprocessed and analyzed resting state functional magnetic resonance imaging data to detect low-frequency inherent signal correlation and concluded that compared with typical development participants, the Rand index (reflecting the similarity between the network organization and the normative network set) of ASD participants was significantly lower [2]. Glaria et al. stated that there are many benefits of compressing real-world graphs, such as improving or enabling visualization in small memory devices, graph query processing, community search, and mining algorithms. This work proposes a novel compact representation for real sparse and clustered undirected graphs. This method uses a fast algorithm to list all the largest cliques and defines a clique graph according to its largest clique [3]. Li et al. showed that the existing vector-based methods of machine learning usually use vector-based features to represent the program, but it is easy to ignore the control information between the basic block and the partition on the path other than the critical path. And they proposed a novel graph-based thread partitioning method to overcome these two bottlenecks. They used graphs to characterize the program, integrated features and control information, and successfully extracted a good partition scheme [4]. Ghasemi said that the problem of power distribution system reconfiguration is a complex optimization process to find a structure with the least loss, which needs to meet the satisfaction of both consumers and the power distribution system company. One of the most important parameters in this regard is to improve the reliability of the system. On the one hand, this parameter improves the satisfaction of electricity consumption, and on the other hand, it improves the economic benefits of power distribution enterprises [5]. Hong H et al. proposed a distribution network reconfiguration method based on a directed graph considering distributed generation. Two reconfiguration scenarios are considered: operating mode adjustment with the goal of minimizing active power loss (case I) and service restoration with the goal of restoring the load to the greatest extent (case II). These two situations are modeled as a mixed integer quadratic programming problem and a mixed integer linear programming problem [6]. Although these studies have reached certain guiding conclusions, there are unavoidable errors, or insufficient optimization effects, insufficient demonstrations, etc., which need to be further improved.

## 3. Distribution Network Reconstruction Model and Graph Theory-Graph Segmentation Method

### 3.1. Image Segmentation Algorithm Based on Graph Theory-Full Variational Approximation of the Ginzburg–Landau Functional of Graph Clustering

The Ginzburg–Landau function is based on the phase transition theory, which combines superconducting phenomena such as quantum mechanics, electrodynamics, and quantum mechanics of superconductors to obtain related nonlinear partial differential equations [7]. Formula (1) expresses the relationship between phase change and phase separation. Letting *S* represent the open subset of *R*^*t*^, the parameter *u* > 0 is the spatial scale:

(1) $$\begin{array}{c} GL\left(v\right)≔\frac{u}{2}\int_{S}{\left|\nabla v\left(a\right)\right|}^{2}dx+\frac{1}{u}\int_{S}W\left(v\left(a\right)\right)dx. \end{array}$$

The form of the Ginzburg–Landau function is a state transition equation, is closely related to the state transition equations such as Allen–Cahn and Chafee–Infante, usually because of the connection between the Ginzburg–Landau function and the total variational seminorm, and is regarded as the second approximation of the total variation, so it can solve the nonsmooth total variation minimization question [8]. The formula used when processing the image is

(2) $$\begin{array}{c} B\left(v\right)=GL\left(v\right)+\lambda f\left(v,v_{0}\right), \end{array}$$

where *f*(*v*, *v*_0_) is the distance function of the reconstructed image *v* and the given image *v*_0_. The statistics of the model are closely related to the physical assumptions. Among them, the parameter *λ* > 0 can control the influence of data fitting on regularization. Applying the *L*^2^ gradient descent method, the partial differential equation at this time can be known:

(3) $$\begin{array}{c} f\left(v,v_{0}\right)={\left\|v-v_{0}\right\|}_{L^{d}\left(S\right)}^{d},d=1,2,\\ vt=-\frac{\beta GL}{\beta v}=u\Delta v-\frac{1}{u}W^{\prime }\left(v\right)-\lambda \frac{\beta f}{\beta v}. \end{array}$$

Because of the existence of the distance function *f(v,v0)*, here we add a forced term *λβf*/*βv*. Since *B*(*v*) is a nonconvex function, there cannot be a unique solution at this time, and the result depends on the initial conditions. The prior information of the image can be used as the initial input of the segmentation algorithm to achieve the goal of more accurate image segmentation in graph theory. Then, the segmented image can be classified with high-dimensional data, and then *I*≔{*a*=(*a*_1_, *a*_2_) ∈ *C*^2^ : 0 ≤ *a*_1_ ≤ *N* − 1; 0 ≤ *a*_2_ ≤ *M* − 1} is set to represent a rectangular image with *K*=*N* × *M* pixels. The image neighborhood of *a* can be represented as set *M*(*a*), *a* ∈ 1:

(4) $$\begin{array}{c} M\left(a\right)≔\left\{b\in 1:\left|a_{1}-b_{1}\right|\leq \varepsilon \text{and}\left|a_{2}-b_{2}\right|\leq \varepsilon \right\}. \end{array}$$

When *ε* ∈ *M*, there are (2*ε*+1) × (2*ε*+1) size pixels centered on *a* in *M*(*a*); for *K* ∈ *M*, we can associate the feature vector *c* ∈ *R*^*K*^ selected by the *a* and *M*(*a*) neighborhoods. Let *X* be the pixel node, *B* the relationship between the vertices mapped to the edge of the graph, *ω* the weight, and *W* the similarity matrix, then

(5) $$\begin{array}{c} \omega \left(a_{z},a_{i}\right)=\omega \left(a_{i},a_{z}\right),\omega \left(a_{z},a_{i}\right)>0,\\ \omega \left(a_{z},a_{i}\right)=\hat{\omega }\left(\gamma \left(a_{z}\right),\gamma \left(a_{i}\right)\right)=\hat{\omega }\left(c_{z},c_{i}\right), \end{array}$$

where *γ* is the characteristic function. At this time, in order to make the symbols consistent, let $\omega \left(a_{z},a_{i}\right)=\hat{\omega }\left(a_{z},a_{i}\right)$, facing the segmentation problem, take the weight of the edge connected to node *x*_*z*_ and the degree *d*_*z*_ of the vertex to obtain a diagonal matrix *D* of *m* × *m*:

(6) $$\begin{array}{c} d_{z}=\sum_{i=1}^{m}\omega_{zi},\\ D=\left[\begin{array}{cccc} d1 & \cdots & \cdots & \cdots \\ \cdots & d_{2} & \cdots & \cdots \\ \vdots & \vdots & \ddots & \vdots \\ \cdots & \cdots & \cdots & d_{m} \end{array}\right]. \end{array}$$

When *X* is used to represent the space of *X*⟶*R* of all functions, *X*⟶*X* is its Laplacian *L*:

(7) $$\begin{array}{c} Lv\left(a\right)=\sum_{b\in X}\omega \left(a,b\right)\left(v\left(a\right)-v\left(b\right)\right),a\in X,\\ L\left(a,b\right)≔\left\{\begin{array}{cc} d\left(a\right), & if\left(a=b\right)\\ 0-\omega \left(a,b\right), & otherwise \end{array}\right). \end{array}$$

The related quadratic form H of *L* can be expressed as

(8) $$\begin{array}{c} H\left(v,Lv\right):\frac{1}{2}\sum_{a,b\in X}\omega \left(a,b\right){\left(v\left(a\right)-\left(b\right)\right)}^{2}. \end{array}$$

The non-negative real eigenvalue of *L* is {*λ*_*z*_}_*z*=1_^*a*^, of which 0=*λ*_1_ ≤ *λ*_2_ ≤ ... ≤ *λ*_*P*_, and under the large-scale limit, *L* can be appropriately scaled to achieve high stability of convergence. At this time, Tulaplas can be normalized:

(9) $$\begin{array}{c} L_{p}≔D^{-1/2}LD^{-1/2}=I-D^{-1/2}WD^{-1/2}. \end{array}$$

At this time, the matrix *L*_*p*_ presents a symmetric state, redefining the discrete Ginzburg–Landau function:

(10) $$\begin{array}{c} GL_{d}\left(v\right)≔\frac{u}{2}H\left(v,L_{p}v\right)+\frac{1}{u}\sum_{a\in X}W\left(v\left(a\right)\right)+\sum_{a\in X}\frac{\chi \left(a\right)}{2}{\left(v\left(a\right)-v_{0}\left(a\right)\right)}^{2},\\ \omega \left(a,b\right)=\exp\left(-{\left\|\gamma \left(a\right)-\gamma \left(b\right)\right\|}^{2}/\sigma^{2}\right),\sigma >0. \end{array}$$

Because this image is an undirected graph, *ω*(*a*, *b*) will be in a symmetrical state, that is, *ω*(*a*, *b*)=*ω*(*b*, *a*). Here, in order to reduce the computational complexity, some feature vectors will be used to construct vectors for graph clustering, and then clustering algorithms will be used to divide their feature vectors to segment the image [9]. The feature vector value is related to the gray or RGB (red, green, blue) intensity value and the texture feature of the neighborhood.

### 3.2. Power Flow Algorithm for Distribution Network Reconstruction

When the distribution network is being reconfigured, when its topological structure is radial, the power flow algorithm can be used to calculate the operation of the distribution network, network losses, and voltage offsets [10]. At present, the power flow algorithms suitable for distribution networks are mainly divided into the Newton method, branch method, and bus method. However, there are certain limitations, and the power flow algorithm is not applicable to the distribution network in some cases. For example, the distribution network and the transmission network have different line parameters, different resistance and reactance ratios, or different numbers of OV nodes. The distribution network will have problems such as frequent line changes and complex structure. Therefore, there will be more power flow algorithms used in the transmission grid than in the distribution network. Based on the increasing attention of the distribution network, improving the convergence, timeliness, and simplicity of the power flow algorithm has become a major goal of the research [11].  Figure 1 is a simple radial distribution network circuit diagram, and its parameters are explained as follows.

The radial distribution network mainly relies on the current quick-break protection at the line outlet, circuit breaker, load switch, and recloser to protect the circuit.

#### 3.2.1. Improving the Basic Principle of the Cow Pull Method

Because it has a better solution effect for nonlinear equations, it is often used in power flow calculations of distribution networks. The Newton-Raphson method voltage polar coordinate formula is

(11) $$\begin{array}{c} {\dot{U}}_{k}=U_{k}<\beta_{k}=U_{k}\left(\cos\;\beta_{k}+i\sin\;\beta_{k}\right). \end{array}$$

Let the distribution network have *x* OL nodes, denoted by 1,2,3, ..., *x*, respectively, and *y* − *x* − 1 PV nodes, denoted by *x*+1, *x*+2, ..., *y* − 1, plus a balance node, then all nodes satisfy

(12) $$\begin{array}{c} \left\{\begin{array}{c} \Delta O_{k}=O_{kr}-O_{k}=O_{kr}-V_{k}\sum_{i=1}^{y}V_{i}\left(W_{ki}\cos\;\beta_{ki}+M_{ki}\sin\;\beta_{ki}\right)=0;k=1,2,...y-1,\\ \Delta L_{k}=L_{kr}-L_{k}=L_{kr}-V_{k}\sum_{i=1}^{y}V_{i}\left(W_{ki}\sin\;\beta_{ki}-M_{ki}\cos\;\beta_{ki}\right)=0;k=1,2,...,x. \end{array}\right) \end{array}$$

According to Taylor's expansion, the modified formula of Newton–Raphson's method can be obtained as

(13) $$\begin{array}{c} \left[\begin{array}{c} \Delta O\\ \Delta L \end{array}\right]=-\left[\begin{array}{cc} S & D\\ F & G \end{array}\right]\left[\begin{array}{c} \Delta \beta \\ U_{H_{2}}^{-1}\Delta U \end{array}\right]. \end{array}$$

The small distance between the actual nodes will only form a small voltage difference between adjacent nodes, so in the calculation, the ground admittance parameter can be ignored. At this time, if *k* ≠ *i*, then

(14) $$\begin{array}{c} S_{ki}\approx \frac{\beta O_{k}}{\beta \theta_{i}}=U_{k}U_{i}M_{ki}\cos\;\theta_{ki},\\ D_{ki}\approx U_{i}\frac{\beta O_{k}}{\beta U_{i}}=-U_{k}U_{i}W_{ki}\cos\;\theta_{ki},\\ F_{ki}\approx U_{i}\frac{\beta L_{k}}{\beta \theta_{i}}=U_{k}U_{i}W_{ki}\cos\;\theta_{ki},\\ G_{ki}\approx U_{i}\frac{\beta L_{k}}{\beta \theta_{i}}=U_{k}U_{i}M_{ki}\cos\;\theta_{ki}. \end{array}$$

If *k*=*i*, then

(15) $$\begin{array}{c} S_{ki}\approx \frac{\beta O_{k}}{\beta \theta_{i}}=-U_{k}\sum_{\begin{array}{c} i=1\\ i\neq k \end{array}}^{y}UiM_{ki}\cos\;\theta_{ki},\\ D_{ki}\approx U_{k}\frac{\beta O_{k}}{\beta U_{k}}=U_{k}\sum_{\begin{array}{c} i=1\\ i\neq k \end{array}}^{y}UiW_{ki}\cos\;\theta_{ki},\\ F_{ki}\approx U_{k}\frac{\beta L_{k}}{\beta \theta_{k}}=U_{k}\sum_{\begin{array}{c} i=1\\ i\neq k \end{array}}^{y}UiW_{ki}\cos\;\theta_{ki},\\ G_{ki}\approx U_{k}\frac{\beta L_{k}}{\beta \theta_{k}}=U_{k}\sum_{\begin{array}{c} i=1\\ i\neq k \end{array}}^{y}UiW_{ki}\cos\;\theta_{ki}. \end{array}$$

The iterative steps of improving the Niu La method are as follows: First, the voltage of the balance node and its phase angle are set, and the parameters of the other node lines are initialized. Then, the calculated parameter values are calculated for active and reactive power corrections, and the accuracy of the power flow calculation is judged until it meets the calculation requirements. Then, the above parameters are substituted into the Jacobian matrix to calculate the voltage amplitude correction amount and phase angle correction amount [12]. Let the number of iterations at this time be *h*, then

(16) $$\begin{array}{c} U_{k}^{\left(h+1\right)}=U_{k}^{\left(h\right)}+\Delta U_{k}^{\left(h\right)};\theta_{k}^{\left(h+1\right)}=\theta_{k}^{\left(h\right)}+\Delta \theta_{k}^{\left(h\right)}. \end{array}$$

Then, the above work is gradually repeated, and the iteration continues.

#### 3.2.2. Distribution Network Reconstruction with DG

The reconstruction step is to initialize various parameters first and number the goals of the distribution network reconstruction and the simplified branches, reinitialize part of the variable value and judge the shape, determine whether it is radial and decide whether to reapply the value, then find the variable of another part of the branch of the distribution network that has been disconnected, and iterate the speed and position. After that, the hierarchical matrix is constructed and combined with the distributed power processing process, and it is pushed back to the power flow calculation before it is completed. Then, the next step is to compare the objective function values to determine the optimal population particle value, continue to iterate and judge the distribution network structure until it is radial and reaches the number of iterations, and finally output the optimal population particle value [13]. The steps are shown in Figure 2.

Here, we will take the IEEE69-node system as an example of distribution network reconstruction. At this time, there are 69 nodes, numbered from 1 to 69. The solid line is the segment switch, and the dashed line is the tie switch. The total system load in this distribution network topology is 3814.6 + *j*2702.2 kVA, and there are 98 iterations of the algorithm. The forward and backward power flow calculations are used to iteratively converge to achieve the minimum network loss. The topology of the distribution network is shown in Figure 3.

In the case of the reconfiguration of the distribution network without distributed power, the initial topology of IEEE69 is that the dashed part denotes the contact switch is off and the solid line denotes the section switch is closed [14]. The reconstruction of the IEEE69-node system without DG is shown in Table 1.

At this time, the network loss of the common algorithm is reduced by 52.98% compared with that before reconstruction, while the algorithm in this paper is reduced by 57.08% compared with that before reconstruction, and the performance is increased by 4.1%, and the effect is better. The network loss of the reconfiguration of the distribution network with distributed power sources is shown in Table 2.

It can be seen that reasonable arrangement of grid-connected locations can reduce network loss. At this time, it has been reduced by 17.27% before reconstruction. After reconstruction, it is reduced by 69.74%. It can be seen that, with the DG power grid, the advantage of its topology is obviously higher than that of power grid without DG. That is, DG reconstruction can improve the voltage quality of the system nodes and improve the operation stability of the distribution network [15].

### 3.3. Distribution Network Fault Recovery Reconstruction Model

Normally, the realization principle of the distribution network fault recovery reconstruction is to use the application layer and the decision-making layer of the distribution network. The control system writes the reconstruction algorithm into the distribution network dispatching system, and the relevant FTU in the distribution network transmits real-time information at the section switch and contact switch. Incorporating data into the SCADA system, the faulty area is located, and here the SCADA system is the control center of the distribution network. Commands are sent to the FTU to isolate the faulty area by operating the switch, the self-healing system is used to generate the structure, optimize algorithm calculations, and control the data, and then the fault area recovery process is performed [16]. In this process, the optimization algorithm is the core part of the distribution network reconstruction, and the voltage, current, power, resistance, frequency, and other states of the distribution network need to be set, and give the range of functions in different states to explore the operation state of the distribution network at this time, and then carry out the optimization search operation [17]. These states include the power grid emergency state, abnormal state, and realm state. The control process of the distribution network is shown in Figure 4.

In the restoration and reconstruction of the distribution network failure, the FTU can quickly locate and isolate the distribution network failure and quickly repair it.

### 3.4. Improved Graph Segmentation Based on Graph Theory BSP-Spark System and Improved JA-BE-JA Algorithm Based on BSP-Spark Cluster

This experiment will be carried out in the environment of a BSP-Spark distributed cluster composed of 4 PCs. Among the PCs, one is used for the main control system with 8 GB of memory, and three are used as slave computing nodes with 4 GB of memory. The software used for compilation is IntelliJ IDEA, and the program used for language writing is Scala. In order to minimize the experimental errors caused by various factors, the machines here will perform tasks one-to-one, and Spark on Yarn will complete resource management and scheduling in the experiment. The storage system is a distributed file system HDFS [18]. It is known that the BSP-Spark system architecture is an M/S architecture, with a complete master-slave relationship, implemented by 1 master node and 3 child nodes. The node deployment diagram is shown in Figure 5.

If it wants to achieve high-performance distributed partitioning, it must optimize the parameters of the BSP-Spark system, such as memory, parallelism, and data skew. Although Spark's calculation is based on memory, there are also algorithms that do not rely on memory. At this time, a caching mechanism needs to be added. In general, the caching method used is spark.executor.memory, and large-scale iterative algorithms need to use a storage mechanism to control the consumption of data access. This article will reduce the set cache to reduce memory consumption, and System.setProperty can just solve this problem [19]. Execution efficiency is closely related to Spark parallelism. Too low parallelism will lead to waste of resources, while too high will reduce efficiency. At this time, spark.default.parallelism is used to optimize the parallelism to ensure the number of tasks. One of the major problems of distributed systems is data skew. During Spark application development, memory overflow exceptions are usually caused. A relatively large amount of graph data corresponds to a relatively small number of node calculations, which will also cause its execution speed to tilt. At this time, shuffle is used to reduce the number of partitions. When small-scale data appear, broadcast variables can be used, and the time interval can be set by spark.speculation.interval [20].

The JA-BE-JA algorithm is a graph partitioning algorithm that combines point partitioning and edge partitioning for load balancing. It comes from the PeerSim environment. Based on the JA-BE-JA algorithm of the BSP-Spark platform, image nodes can be processed asynchronously on a regular basis, and a node only interacts with a small random range of adjacent nodes. The information dissemination between nodes is only through the edges of the image and is based on memory sharing. Its vertices correspond to a single node host and process threads independently. The image dataset input by the improved JA-BE-JA algorithm is only in *G(V,E)* format, and the image data need to be preprocessed before dividing. Preprocessing includes split-transform-storage, and graph data cleaning uses transformation and action operators to generate new edge RDDs and vertex RDDs from the data source. The algorithm flow is shown in Figure 6.

The edge segmentation and point segmentation of the JA-BE-JA algorithm are realized by the Graph.partitionBY operator, and the mixed sampling method is preferred for the sampling strategy.

## 4. Results and Analysis

### 4.1. Experimental Results and Analysis

Here, we will collect the edge cuts of the JA-BE-JA algorithm based on the BSP-Spark platform in the distributed segmentation of 4 image datasets with data sizes ranging from small to large, then collect the edge cuts of the JA-BE-JA algorithm based on the BSP-PeerSim platform in the same dataset, and collect them after 1200 supersteps to ensure the accuracy of the experiment [21–23]. The experimental results are shown in Figures 7 and 8.

It can be seen that the size of the vertices and edges of the 4elt graph is small, and the difference in the number of edge cuts is small, while the size of the vibrobox graph is larger, and the trend of the number of edge cuts gradually tends to be flat.

Next, the improved annealing simulation algorithm is analyzed. It is known that the improved BSP-Spark algorithm has better load in large-scale graph segmentation, but it is easy to form a local optimal state. Therefore, this article will propose an improved annealing algorithm based on BSP-Spark and perform performance testing, taking two parameters *u* and *v* for performance measurement; let *u* be the parameter of the edge cut problem of the improved JA-BE-JA algorithm and be the system energy function value. The relationship between *u* and JA-BE-JA algorithm in the original BSP-PeerSim and BSP-Spark environments is shown in Figure 9.

It can be seen that the improved annealing simulation algorithm has a smaller edge cut when *u* = 2. This is because when this parameter is greater than 1, graph partitioning can reduce the number of communication edges without damaging the original topological structure of the graph and reduce information propagation and iteration time. When the parameter *u* = 3, the consumption of information dissemination will increase due to the reduction of the total effect value of the graph. This situation will become more serious as the parameter *u* increases. The improved annealing model algorithm can reduce the consumption when *u* = 2 and reduce the probability of the local optimal problem of the JA-BE-JA algorithm. Let *v* be the cooling coefficient, which can represent the cooling rate, and the relationship between it and the edge cut number of the JA-BE-JA algorithm is shown in Figure 10.

It can be seen from the Figure 10 that based on the original BSP-PeerSim environment, the number of edge cuts increases with the increase of the parameter *v*, and *v* can represent the equalization effect of the number of exchanges and the quality of graph division. That is to say, the greater the number of exchanges, the longer the convergence time, and the information dissemination consumption will increase. Based on the BSP-Spark environment, the edge cut value of the obvious graph has robust stability for the parameter *v*.

In the improved data migration algorithm, local optimization problems can be avoided, and random functions can be used to reduce the number of communication edges. At this time, using different datasets for testing, it can be seen that a 4-way partition will cause 76.3% of the vertex data to migrate, and only 23.7% of the data moved to different partitions.

### 4.2. Improved Graph Theory and Graph Segmentation Method Cited into the Distribution Network Calculation Examples and Result Analysis

Here, we will use the improved JA-BE-JA algorithm to calculate the distribution network example. The 16-busbar system of the distribution network has 3 tie switches and 3 feeders, as shown in Figure 11.

The tie switch is closed, the weighting operation is performed on the 16-bus distribution system, the eigenvector is solved by the spectral division algorithm, and the critical edge of the above-mentioned distribution system and the node of division 1 are removed [24].  Figure 12 is available.

The above figure is a subgraph based on the feature evaluation value after the first scoring and sorting, and its feature evaluation value is shown in Figure 13 at the same time as the feature evaluation value after the second scoring and ranking. The distribution network nodes are divided into groups: group 1 is {1,2,4,5,6,7,8,9,11,12}, group 2 is {3,10,13,14,15,16}, which is recorded as division 1, and the rest of the system needs to be divided into two using the improved JA-BE-JA algorithm, that is, division 2: {1,4,5,6,7,11} and division 3: {2,8,9,12}, and Figure 13 can be obtained.

It can be seen that the final reconstruction result of the distribution network is to close the tie switch between nodes 10 and 14, close the tie switch between 5 and 11, open the section switch between 8 and 10, turn on the segment switch between 9 and 11, and use the improved JA-BE-JA algorithm graph theory to divide the network loss to 454.3 KW. The initial network loss is 508.6 KW, and the network loss is reduced by 10.68%. The power distribution system is often of large-scale and widely distributed, and there are multiple feeders. It can be seen that this algorithm is still applicable in large-scale distribution networks, reducing the burden of power flow calculation, reducing the network loss, and also solving the problem of local optimization.

## 5. Discussion

This article focuses on the analysis of large-scale distribution network reconstruction with graph theory and graph partitioning algorithms. Image segmentation based on graph theory has been developed in many fields and has made indelible contributions in medicine and neurology [25]. This article first describes many advantages of graph theory and graph segmentation technology in the application of distribution networks and then describes the research methods of graph theory and graph segmentation and distribution networks. For example, the image segmentation method based on graph theory-full variational approximation of the Ginzburg–Landau functional of graph clustering uses quantum mechanics, superconductor, electrodynamics, and other phenomena to derive relevant formulas, divides the feature vector through the clustering algorithm, and performs image segmentation. For example, for the power flow algorithm of distribution network reconstruction, the radial circuit diagram is given in this article, and the power flow algorithm is used for calculation according to the topology of the distribution network. In this paper, the improved Niu pull method is used to improve convergence, timeliness, etc., phase angle correction and voltage correction are carried out, the distribution network reconstruction with DG is proposed, and the optimal value of the population particles is repeatedly iterated. The IEEE69 example is used to show the situation, and the forward and backward power flow calculations are used to iteratively converge to achieve the minimum network loss. It also describes the fault recovery model of the distribution network, using the application layer, decision-making layer, and control system of the distribution network to write the reconstruction algorithm into the distribution network dispatching system. The faults of the distribution network are quickly located and isolated through the FTU, and quickly repaired. Finally, the graph theory algorithm and the performance of the improved JA-BE-JA algorithm are tested through experiments, and they are applied to the distribution network, and the relationship between each partition and the JA-BE-JA algorithm is compared. Substituting the parameters into the test, it can be seen that a 4-way partition will cause migration of a large number of vertex data, and migration of only a small part of the data to different partitions. Finally, a 16-bus distribution system example is used for testing, and the improved JA-BE-JA algorithm can reduce the loss by 10.68% compared with the previous one, and it can be applied to a multifeeder system, that is, the large-scale distribution network, which reduces the power flow calculation. It can also reduce network loss and prevent local optimization. It can be obtained that this improved algorithm can be better applied in large-scale distribution networks.

## 6. Conclusions

In the analysis of large-scale distribution network reconstruction with graph theory and graph partitioning algorithms, it is known that based on the BSP-Spark environment, the improved algorithm has robust stability and can avoid the problem of local optimization. A 4-way partition caused 76.3% of the vertex data migration, and only 23.7% moved to a different partition. The improved JA-BE-JA algorithm is also more obvious for the optimization of the distribution network. Using the improved JA-BE-JA algorithm with graph theory and graph division, the network loss is 454.3 KW, the initial network loss is 508.6 KW, and the network loss is reduced by 10.68%. In addition, the improved algorithm can effectively increase the number of edge cuts and the number of vertices exchanged on the distributed clusters. It is much more effective than the traditional graph segmentation algorithm in the processing of large-scale distribution networks.

## Figures and Tables

**Figure 1:** Circuit diagram of a typical radial distribution network.

**Figure 2:** Distribution network reconstruction algorithm flow.

**Figure 3:** IEEE69 distribution network node topology.

**Figure 4:** Distribution network control process.

**Figure 5:** Node deployment.

**Figure 6:** Improved JA-BE-JA algorithm flow.

**Figure 7:** Relationship between the two partitions of 4elt graph and vibrobox and the edge cut number of the JA-BE-JA algorithm.

**Figure 8:** Relationship between the two partitions of Twitter and web-Google and the edge cut number of the JA-BE-JA algorithm.

**Figure 9:** Relationship between *u* and JA-BE-JA algorithm in the original BSP-PeerSim and BSP-Spark environments.

**Figure 10:** Relationship between v and the JA-BE-JA algorithm edge cut number.

**Figure 11:** Bus distribution system.

**Figure 12:** Subgraph after halving processing.

**Figure 13:** Comparison of feature evaluation values after the first and second sorting.

**Table 1:** Distribution network reconstruction results without DG grid connection.

State	Disconnect switch position	Lowest node voltage	Network loss (kW)
Before reconstruction	27/70/71/72/73	0.912	231.25
Ordinary algorithm	13/43/50/71/72	0.951	108.74
The algorithm of this paper	14/44/50/71/72	0.946	99.26

**Table 2:** Distribution network reconstruction results when DG is connected to the grid.

State	Disconnect switch position	Lowest node voltage	Network loss (kW)
Before reconstruction	27/70/71/72/73	0.912	231.25
Before reconstruction (including DG)	27/70/71/72/73	0.931	191.32
After reconstruction (including DG)	13/46/51/71/72	0.962	69.98

## Data Availability

The data used to support the findings of this study are available from the author upon request.
